# Taurine-Upregulated Gene 1 Attenuates Cerebral Angiogenesis following Ischemic Stroke in Rats

**DOI:** 10.1155/2022/1037525

**Published:** 2022-10-25

**Authors:** Fei Li, Jun-Hua Yu, Hong-Xiang Jiang, Hui-Kai Zhang, Qiang Cai, Zai-Ming Liu, Ming-Chang Li, Qian-Xue Chen

**Affiliations:** ^1^Department of Neurosurgery, Renmin Hospital of Wuhan University, Wuhan 430060, Hubei, China; ^2^Ezhou Central Hospital, Ezhou 436000, Hubei, China

## Abstract

**Objective:**

Angiogenesis is one of the therapeutic targets of cerebral infarction. Long noncoding RNAs (lncRNAs) can regulate the pathological process of angiogenesis following ischemic stroke. Taurine-upregulated gene 1 (TUG1), an lncRNA, is correlated to ischemic stroke. We intended to determine the effect of TUG1 on angiogenesis following an ischemic stroke.

**Materials and Methods:**

Middle cerebral artery occlusion (MCAO) was adopted to build a focal ischemic model of the rat brain, and pcDNA-TUG1 and miR-26a mimics were injected into rats. Neurological function was estimated through modified neurological severity scores. The volume of focal brain infarction was calculated through 2,3,5-triphenyltetrazolium chloride staining. The level of TUG1 and miR-26a was measured by PCR. The expression of vascular endothelial growth factor (VEGF) and CD31 was checked using immunohistochemistry and western blot. The correlation between miR-26a and TUG1 was verified through a luciferase reporter assay.

**Results:**

TUG1 increased noticeably while miR-26a was markedly reduced in MCAO rats. Overexpression of miR-26a improved neurological function recovery and enhanced cerebral angiogenesis in MCAO rats. TUG1 overexpression aggravated neurological deficits and suppressed cerebral angiogenesis in MCAO rats. Bioinformatics analysis revealed that miR-26a was one of the predicted targets of TUG1. Furthermore, TUG1 combined with miR-26a to regulate angiogenesis. TUG1 overexpression antagonized the role of miR-26a in neurological recovery and angiogenesis in MCAO rats.

**Conclusions:**

TUG1/miR-26a, which may act as a regulatory axis in angiogenesis following ischemic stroke, can be considered a potential target for cerebral infarction therapy.

## 1. Introduction

Ischemic stroke, which is caused by a blockage in one or more arteries that supply blood to the brain, is by far the most common subtype of stroke [1]. Although considerable research has been conducted in the past [2–6], there are few effective therapies for cerebral ischemia. Therefore, the development of effective therapies for ischemic stroke remains an unmet health care need.

Angiogenesis is conducive to the improvement of functional outcomes after ischemic strokes and is consequently an important therapeutic target for cerebral infarction [7–9]. Angiogenesis is a process in which vascular endothelial cells undergo a series of pathophysiological changes to sprout new blood vessels under the coregulation of angiogenic promotors and angiogenesis inhibitors. However, the mechanism of angiogenesis after ischemic stroke has not been well clarified.

Studies have borne out claims that long noncoding RNAs (lncRNAs) play a key role in angiogenesis following ischemic stroke [10, 11]. As an lncRNA, taurine-upregulated gene 1 (TUG1) is widely expressed in many tissues. More recently, it was reported that TUG1 can regulate angiogenesis in diverse clinical scenarios [12, 13]. Abdelaleem et al. [14] found that serum lncRNA TUG1 might be a useful novel molecular biomarker for diabetes complicated by a stroke. Earlier researches suggested that TUG1 may have a vital role in the pathological changes after cerebral infarction [15, 16]. However, the role and mechanism of TUG1 on angiogenesis following cerebral infarction remain hazy. Studies clarified that miR-26a can promote angiogenesis under various physiological and pathological conditions [17, 18]. Previous reports have displayed that lncRNAs had considerable impact on miRNA-mediated gene downregulation or upregulation by playing the role of competing endogenous RNAs or miRNA sponges [19–21]. Using bioinformatics tools, we detected the binding site for miR-26a in TUG1. We aim to describe the potential regulatory role of TUG1 in angiogenesis following cerebral ischemia via modulating miR-26a.

## 2. Materials and Methods

### 2.1. Animals

All procedures using laboratory animals were permitted by the Ethics Committee (Animal) of Renmin Hospital of Wuhan University (Approval No. WDRM2020-K071). Sprague Dawley rats (230-270 g, male) used in our research were provided by the Experimental Animal Center of Wuhan University.

### 2.2. Rat Model of Cerebral Ischemia

The right middle cerebral artery occlusion (MCAO) model was established as previously described [22]. During the operation of the MCAO, the cerebral blood flow of rats was monitored using a Laser Doppler Flowmeter (Perimed, Sweden) to evaluate the successful occlusion of the middle cerebral artery, which was defined as a decrease of more than 70% in cerebral blood flow. The temperature was maintained at 37 ± 0.5°C until the rats woke up. The signs of successful surgery are defined as follows: homolateral Horner's sign, weakened grasping ability of the contralateral forelimb, and uncontrollably rotating or tilting to left. The same operation procedure was applied to the rats in the sham group without occlusion of cerebral artery.

### 2.3. RNA Oligonucleotides and Plasmid Construction

The design and construction of recombinant plasmids, including pcDNA-NC (negative control) and pcDNA-TUG1, were done by Genechem (Shanghai, China). miR-26a mimics and mimics-NC were all from RiboBio (Guangzhou, China).

### 2.4. Grouping and Treatment in the MCAO Model

All surviving rats were randomly grouped as follows (*n* = 6): sham group, MCAO group, MCAO+pcDNA-TUG1 group (performing intracerebroventricular injection of TUG1 overexpression plasmid), MCAO+pcDNA-NC group (performing intracerebroventricular injection of empty plasmid), MCAO+miR-26a mimics group (receiving tail vein injection of miR-26a mimics), MCAO+mimics-NC group (receiving tail vein injection of mimics-NC), MCAO+miR-26a mimics+pcDNA-TUG1 group (injected with TUG1 overexpression plasmid and miR-26a mimics), and MCAO+miR-26a mimics+pcDNA-NC group (injected with empty plasmid and miRNA mimics).

The in vivo administration of pcDNA-TUG1 and pcDNA-NC was performed as described previously [23]: one day before MCAO, rats were fixed after anesthesia and injected in the right lateral ventricle (the drilling position is 0.8 mm behind bregma, 1.5 mm to the right of midline; the puncture depth is 4.5 mm from the skull surface), with 5 *μ*l of the plasmid. miR-26a mimics or negative controls were injected through the tail vein as previously reported [24].

### 2.5. Neurological Function Assessment

The neurological function in rats was appraised using modified neurological severity scores (mNSS), 1, 3, and 7 days after MCAO. The score was completed by two investigators who were blind to the experiment. The score of neurological function ranged from 0 to 18 (0 means normal score, while 18 represents the maximal deficit score), in which a higher score indicates a more severe neurological deficit.

### 2.6. Infarct Volume Testing

On the seventh day after MCAO, all rats were killed and specimens were collected for further analysis. The frozen brains were sliced into continuous slices (approximately 2 mm thick, coronal). 2,3,5-Triphenyltetrazolium chloride (TTC) (2%) was used to stain the sections (37°C, 15 minutes); then, the sections were fixed in paraformaldehyde at 4°C all night. The volume of cerebral infarction was quantified through a computerized image analyzer [25].

### 2.7. Cell Culture and Treatment

HEK-293T cells were presented by the Central Laboratory, Renmin Hospital of Wuhan University. The complete medium for culturing cells contains DMEM medium with fetal bovine serum (10%) and penicillin-streptomycin (concentration, 100 U/mL), under the condition of 5% CO_2_ humidified atmosphere at 37°C.

### 2.8. Luciferase Reporter Assay

By using Lipofectamine 2000 reagent (Invitrogen, CA, Carlsbad, USA) based on the manual, pmirGLO-TUG1-3′UTR wild type (pmirGLO-TUG1-WT) or pmirGLO-TUG1-3′UTR mutant (pmirGLO-TUG1-MUT) was transfected into HEK-293T cells, into which miR-26a mimics or mimics-NC were cotransfected, respectively. Luciferase activity was tested 48 hours after transfection.

### 2.9. Immunohistochemistry (IHC)

The brain tissue samples of rats were fixed in paraformaldehyde (concentration of 4%), paraffin-embedded, and then sectioned at 4 *μ*m. After dewaxing and hydration of sections, the slices were treated for 20 minutes with 3% H_2_O_2_ solution. The sections were placed in citrate buffer (concentration, 10 mmol/l) and heated by microwave for 30 minutes to achieve antigen retrieval. Then, the sections were blocked using normal goat serum. Following that, the primary antibody and the secondary antibody were added successively for incubation. The cerebral histological sections were then washed and incubated in peroxidase substrate solution. All stained slices were observed through an optical microscope after reaching the required stain intensity. The positive staining of VEGF and CD31 was light to dark brown, mainly located in the cytoplasm and cell membrane. CD31 staining was performed as an indicator of microvessel density (MVD). The MVD values were calculated as per the criteria proposed by Weidner et al. [26].

### 2.10. qRT-PCR

Using a TRIzol reagent (Invitrogen, Shanghai, China), we isolated RNA from brain tissues in accordance with the instructions. The expression levels of the genes were quantified by qRT-PCR technology. The 2^-*ΔΔ*CT^ calculation was adopted to work out the relative quantities of subject genes. U6 RNA served as the internal control for miR-26a. For TUG1 and VEGF, the internal control was GAPDH. The following are the primer sequences of these genes:

- TUG1: forward 5′-ACCCTGTGGAGTACCCAGGA C-3′, reverse 5′-GGGTTGTTCTCTAGAGTTGCTGG-3′
- GAPDH: forward 5′-CGCTAACATCAAATGGGGTG-3′, reverse 5′-TTGCTGACAATCTTGAGGGAG-3′
- miR-26a: forward 5′-TGCAAGTAATCCAGGATAGGCT-3′, reverse 5′-CTCAACTGGTGTCGTGGAGTC-3′
- VEGF: forward 5′-ATGTGTGTCCGTCTACAGATGT-3′, reverse 5′-GGAAGTGTGATTGGCAAAACTGA-3′
- U6: forward 5′-CCTGCTTCGGCAGCACAT-3′, reverse 5′-AACGCTTCACGAATTTGCGT-3′

### 2.11. Western Blot

Proteins were isolated from rat brain samples and separated using SDS-PAGE. The proteins were then transferred to polyvinylidene difluoride membranes and incubated with their respective primary antibodies (4°C, overnight). After washing, the corresponding secondary antibody was used to examine the bound antibodies. GAPDH served as the internal control.

### 2.12. Statistical Analysis

SPSS 20.0 was used to perform statistical calculation. Data are shown as the mean ± standard deviation (SD) for measurement variables. Differences between the two groups were measured using Student's *t*-test. Differences among three or more groups were analyzed using one-way ANOVA with Bonferroni's post hoc test. *P* < 0.05 was accepted as indicative of significant differences.

## 3. Results

### 3.1. TUG1 Is Upregulated and miR-26a Is Downregulated following Ischemic Stroke

The relative level of TUG1 and miR-26a in samples after cerebral infarction was detected by qRT-PCR. Our data indicated that the relative ratio of TUG1 was markedly higher in MCAO rats than in control rats (Figure 1(a)). Our results also announced that miR-26a decreased largely in MCAO rats (Figure 1(b)).

### 3.2. miR-26a Improves Neurological Function Recovery and Promotes Angiogenesis in MCAO Rats

Considering the significant downregulation of miR-26a in response to ischemia in vivo, we examined the effects of miR-26a on ischemic stroke injury through artificially overexpressing miR-26a. After injection of miR-26a mimics, the level of miR-26a in rat brain tissues increased substantially (Figure 2(a)). There was no significant difference in mNSS between the MCAO group and MCAO+miR-26a mimic group on the first day after MCAO. However, in the MCAO+miR-26a mimics group, mNSS improved obviously compared with the MCAO group on the third and seventh day after operation (Figure 2(b)). TTC staining revealed that the area of cerebral infarction was effectively reduced after injection of miR-26a mimics (Figure 2(c)). qRT-PCR analysis of the angiogenesis-related gene VEGF confirmed the boosting effect of miR-26a on cerebral angiogenesis (Figure 2(d)). Results of IHC exhibited that, after injection of miR-26a mimics, the level of VEGF and MVD in the brain tissues of MCAO rats was remarkably increased (Figures 2(e) and 2(f)). Furthermore, western blot analysis also revealed higher expression of cytoplasmic VEGF and CD31 in the miR-26a mimic group (Figure 2(g)).

### 3.3. TUG1 Overexpression Aggravates Infarction Volume and Neurological Function Defects in MCAO Rats

As exhibited in Figure 3(a), the expression of TUG1 was substantially upregulated in the MCAO+pcDNA-TUG1 group, compared with that derived from the pcDNA-NC-treated rats. Compared with those in the MCAO+pcDNA-NC group, rats in the MCAO+pcDNA-TUG1 group exhibited marked neurological dysfunction on the third and seventh day after MCAO (Figure 3(b)). Results of TTC staining showed that after being injected with the liposome pcDNA-TUG1, the area of cerebral infarction was effectively increased (Figure 3(c)). It was also exhibited that TUG1 overexpression significantly inhibited VEGF mRNA expression (Figure 3(d)). Results of IHC exhibited that upregulation of TUG1 remarkably inhibited the expression level of VEGF and MVD in the ischemic cerebral cortex of MCAO rats (Figures 3(e) and 3(f)). Western blot analysis also revealed lower expression of cytoplasmic VEGF and CD31 in the TUG1 overexpression group (Figure 3(g)).

### 3.4. TUG1 Targets miR-26a And Negatively Regulates Its Expression

To determine the interaction of miR-26a and TUG1, we used starBase. As shown in Figure 4(a), the results from starBase indicated that miR-26a was a potential target of TUG1. Subsequently, a luciferase reporter assay was performed. We found that after cotransfection with miR-26a mimics, luciferase activity was markedly reduced in HEK-293T cells transfected with WT-TUG1 but not MUT-TUG1 (Figure 4(b)). Next, we adopted qRT-PCR to confirm whether miR-26a could be negatively regulated by TUG1. The results revealed that injection of pcDNA-TUG1 noticeably decreased the relative level of miR-26a in brain samples (Figure 4(c)).

### 3.5. TUG1 Regulates Neurological Functional Recovery and Cerebral Angiogenesis in MCAO Rats via miR-26a

Based on the above results, we hypothesized that TUG1 affects ischemic damage and angiogenesis via downregulation of miR-26a. As shown in Figure 5(a), the injection of pcDNA-TUG1 attenuated the effect of miR-26a on improving neurological function in rats on the third and seventh day after MCAO. In addition, TUG1 overexpression partly reversed the activation of VEGF mRNA expression by miR-26a in MCAO rats (Figure 5(b)). In Figures 5(c)–5(e), it was found that TUG1 overexpression can also reverse the intensification of miR-26a on VEGF protein expression. Consistent with this observation, MVD in the ischemic cerebral cortex of MCAO rats overexpressing miR-26a was also decreased by TUG1. These results indicated that TUG1 regulated angiogenesis via regulating miR-26a.

## 4. Discussion

This study explored the possible regulatory effect and potential mechanisms of TUG1 on angiogenesis following ischemic stroke. After the establishment of the MCAO model, we found that TUG1 was upregulated in rat brains. Overexpressing TUG1 could aggravate neurological deficits and suppress cerebral angiogenesis in MCAO rats. Furthermore, TUG1 negatively regulated miR-26a expression and attenuated the role of miR-26a in improving neurological function and angiogenesis in MCAO rats.

Previous studies have demonstrated that TUG1 plays an essential role in various ischemic stroke-related procedures [27]. They have also confirmed that the serum TUG1 level of diabetic patients with ischemic stroke is significantly higher than that of diabetic patients without ischemic stroke, and the serum TUG1 level is positively correlated with the NIHSS score of the patients [14]. TUG1 rs2240183 may be used as a new biomarker to predict the short-term prognosis of patients with ischemic stroke [28]. In acute ischemic stroke, lncRNA TUG1 can enhance neuronal damage mediated by ERK12 signal pathway [29]. In addition, TUG1 can sponge miR-204-5p to aggravate ischemia-reperfusion injury of neurons [30]. It is widely known that angiogenesis, which is a multistep process, serves as an important protective mechanism against cerebral infarction [31]. However, the potential effect of TUG1 on angiogenesis after ischemic stroke is not fully clarified. In this research, we observed that TUG1 aggravated infarction volume and neurological deficit in MCAO rats. VEGF, as is well-known, can promote proliferation and differentiation of vascular endothelial cells, which plays a key role in angiogenesis [32]. We also found that TUG1 markedly decreased MVD and expression of VEGF protein and mRNA in the ischemic cerebral cortex of MCAO rats. These findings suggested that TUG1 can repress angiogenesis following cerebral ischemia in rats.

In our study, miR-26a was downregulated in MCAO rats, displaying changes contrary to TUG1. A study by Wang et al. demonstrated that miR-26a promoted angiogenesis via upregulating VEGF by activating the PI3K/Akt signaling pathway [33]. Similarly, our research also showed that miR-26a promotes the protein and mRNA expression of VEGF and CD31. Previous researches have exhibited that lncRNAs may serve as competing endogenous RNAs (ceRNAs) via their competition for miRNA binding, decreasing the miRNA expression levels, which are accessible for downstream mRNA [34]. Therefore, we investigated the correlation between TUG1 and miR-26a. Using bioinformatics prediction and luciferase reporter assay, we identified that miR-26a can bind to TUG1 directly. Further researches revealed that TUG1 could effectively downregulate the expression of miR-26a and abolish the promoting role of miR-26a in angiogenesis following cerebral infarction. To summarize, our study indicates that TUG1 inhibited angiogenesis following cerebral infarction by negatively modulating the expression of VEGF through sponging miR-26a.

Nonetheless, our research has certain limitations. The main limitation is that it is only an in vivo experiment without the verification of clinical cases. The role and mechanism of TUG1 in angiogenesis following ischemic stroke have not been verified in human tissue samples. More research is needed in the future.

## 5. Conclusions

The current research demonstrated that lncRNA-TUG1/miR-26a, which can act as a regulatory axis in angiogenesis following ischemic stroke, can be provided as a potential target for cerebral infarction therapy.

## Figures and Tables

**Figure 1:** TUG1 is overexpressed, and miR-26a is underexpressed in MCAO rats. (a) TUG1 expression in brain tissues after ischemic stroke. (b) miR-26a relative level in brain samples following cerebral infarction. Data are shown as the mean ± SD (*n* = 6 for each group). ^∗∗∗^*P* < 0.001.

**Figure 2:** Overexpression of miR-26a improves neurological function recovery and promotes cerebral angiogenesis in MCAO rats. (a) Modulation of miR-26a levels by scramble RNA or miR-26a mimics in MCAO rats. (b) Neurological function of MCAO rats evaluated by mNSS. (c) Volume of cerebral ischemia. (d) Relative VEGF mRNA levels in MCAO rats after injection of miR-26a mimics. (e, f) Expression of VEGF and CD31 detected by IHC (400x). (g) Protein expression levels of VEGF and CD31 detected by western blot. Data are shown as the mean ± SD (*n* = 6 for each group). ^∗∗∗^*P* < 0.001, compared with the sham group; ^###^*P* < 0.001, compared with the mimics-NC group.

**Figure 3:** TUG1 aggravates neurological deficits and inhibits cerebral angiogenesis. (a) Expression of TUG1 in various groups of rats. (b) Neurological function of MCAO rats evaluated by mNSS. (c) Infarction volume in rats with focal cerebral ischemia detected by TTC staining. (d) Relative VEGF mRNA levels in MCAO rats after injection of pcDNA-TUG1. (e, f) Expression of VEGF and CD31 detected by IHC (400x). (g) Protein expression levels of VEGF and CD31 detected by western blot. Data are shown as the mean ± SD (*n* = 6 for each group). ^∗∗∗^*P* < 0.001, compared with the sham group; ^#^*P* < 0.05, compared with the pcDNA-NC group; ^##^*P* < 0.01, compared with the pcDNA-NC group; ^###^*P* < 0.001, compared with the pcDNA-NC group.

**Figure 4:** TUG1 binds to miR-26a and regulates the relative level of miR-26a. (a) Binding site of TUG1 on miR-26a predicted using bioinformatics software. (b) Luciferase reporter assay of TUG1 and miR-26a (*n* = 3). (c) miR-26a expression in MCAO rats injected with pcDNA-NC or pcDNA-TUG1 (*n* = 6 for each group). Data are shown as the mean ± SD. ^∗∗∗^*P* < 0.001, compared with the mimics-NC group; ^∗∗∗^*P* < 0.001, compared with the sham group; ^###^*P* < 0.001, compared with the pcDNA-NC group.

**Figure 5:** TUG1 antagonizes the promotion of VEGF by miR-26a to regulate neurological functional recovery and cerebral angiogenesis in MCAO rats. (a) Neurological function of MCAO rats in various treatment groups. (b) Relative VEGF mRNA levels in MCAO rats in various groups. (c) Images from IHC photographs of VEGF in various groups (400x). (d) Expression of CD31 and count of MVD in brain samples of MCAO rats in various groups. Magnification of the microphotograph, ×400. (e) VEGF and CD31 protein expression among each group. Data are shown as the mean ± SD (*n* = 6 for each group). ^∗∗∗^*P* < 0.001, compared with the mimics-NC group; ^##^*P* < 0.01, compared with the miR-26a mimics+pcDNA-NC group; ^###^*P* < 0.001, compared with the miR-26a mimics+pcDNA-NC group.

## Data Availability

The data supporting the conclusions of this study are available from the corresponding author.
